The article "Comprehensive Analysis of the Expression of TGF-β Signaling Regulators and Prognosis in Human Esophageal Cancer" was published in 2021. Journal: Comput Math Methods Med.

# Comprehensive Analysis of the Expression of TGF-*β* Signaling Regulators and Prognosis in Human Esophageal Cancer

**DOI:** 10.1155/2021/1812227

**Published:** 2021-10-23

**Authors:** Wei Song, Wei-Jie Dai, Meng-hui Zhang, Han Wang, Xiao-Zhong Yang

**Affiliations:** Department of Gastroenterology, The Affiliated Huai'an No.1 People's Hospital of Nanjing Medical University, Huai'an 223300, China

## Abstract

More and more evidences show that TGF-*β* has a crucial role in tumor initiation and development. However, the mechanism of the TGF-*β* signal regulator in esophageal cancer (EC) is still unclear. Here, we use a variety of bioinformatics methods to analyze the expression and survival data of TGF-*β* signal regulators in patients with EC. We extracted the expression of the S-TGF-*β* signal regulator from The Cancer Genome Atlas (TCGA). The cBioPortal database was used to assess the frequency of genetic variation. The TGF-*β* signal regulator is expressed in EC and normal tissues. The objective is to use the Kaplan-Meier plotter database to investigate the prognostic value of TGF-*β* signal regulators in cancer patients. The DAVID and clusterProfiler software package were used for functional enrichment analysis. We found that patients with TGF-*β* signaling mutations have shorter overall survival, disease-free survival, disease-specific survival, platinum overall survival, and platinum-free progression survival. We found that compared with the noncancerous tissues of patients with EC, ZFYVE9, BMPR1B, TGFB3, TGFBRAP1, ACVRL1, TGFBR2, SMAD4, SMAD7, ACVR2A, BMPR1, and SMAD9 were significantly downregulated in tumor tissues, while ACVR1 and Smad1 were significantly upregulated in tumor samples. Univariate survival analysis showed that ACVR1, TGFBR3, TGFBRAP1, BMPR1A, SMAD4, and TGFBR2 were positively correlated with overall survival (OS) prolongation. In addition, TGF-*β* signal transduction regulators could be divided into two classes. Subclass 1 was involved in regulating cell adhesion, PI3K-Akt signaling, and Rap1 signaling. Subclass 2 was related to regulating angiogenesis and PI3K signaling. In short, all members of TGF-*β* signal regulators can be used as biomarkers to predict the prognosis of patients with EC.

## 1. Background

Esophageal cancer (EC) is the eighth most common malignant tumor in the world, posing a great threat to public health [1, 2]. Esophageal squamous cell carcinoma (ESCC) has the characteristics of strong invasiveness, high metastasis rate, and poor prognosis [3]. It is reported to be the most common histological subtype of EC, accounting for nearly 80% of all EC incidences [4]. After 4 or 5 years of diagnosis, the 5-year survival rate of patients with EC is only 15-25% [4]. There is increasing evidence that some genetic and epigenetic changes contribute to the tumorigenesis of ESCC [5]. It is of great significance to find new therapeutic targets for ESCC.

The article "Comprehensive Analysis of the Expression of TGF-β Signaling Regulators and Prognosis in Human Esophageal Cancer" was published in 2021. Journal: Comput Math Methods Med.

TGF-*β* exerts its function in human cells. In a typical signaling, a TGF-*β* ligand binds to a heterotetrameric receptor complex including TGFBR1 and TGFBR2 [6]. Then, the ligand and receptor complex phosphorylated and activated downstream SMAD2/3, which is a component of a transcription factor [7]. The Smad complex then cooperates with other regulators to direct transcription activation and regulate multiple downstream mechanisms [8]. However, Smad7 could also suppress the activation of TGF-*β*/Smad signaling through competitively binding to TGFBR1 [9]. In addition, the TGF-*β* pathway could crosstalk with Rho, PI3K, and MAPK signaling to promote EMT, invasion, and angiogenesis [10]. Previous studies had demonstrated the important roles of TGF-*β* in human cancers. For instance, TGF-*β* modulates the cell cycle through the transcriptional regulation inhibitors p15INK4 and p21CIP1 [11]. In addition, the TGF-*β*/Smad axis also promotes cell stemness and mesenchymal transformation by upregulating multiple gene expression, such as Snail and Vim [12]. Understanding the expression profile and potential functions of TGF-*β* signaling could provide novel clues to identify novel treatment markers for esophageal cancer.

To the best of our knowledge, a comprehensive analysis has yet to be applied to clarify the role of TGF-*β* signaling regulators in EC. Based on various bioinformatics databases, this study detected the RNA levels and mutation status of the TGF-*β* signal regulator in EC and predicted the potential functions of these regulators in EC.

## 2. Materials and Methods

### 2.1. TCGA Database

TCGA included the RNA sequence data of human genes in more than 30 cancer types. The expression profile of the TGF-*β* signal regulator is retrieved from TCGA database, and the clinicopathological information of EC patients are also downloaded from this database [13]. The receiver operating characteristic (ROC) [14] curve assesses the diagnostic value of the TGF-*β* signal regulator in EC patients.

### 2.2. cBioPortal Database

cBioPortal (https://www.cbioportal.org/) provides large-scale cancer genome data and was used to evaluate the frequency of TGF-*β* signal regulator mutations in EC patients [15].

### 2.3. Analysis of Correlation and Function Enrichment of the TGF-*β* Signal Regulator

The Corrplot [16] software package was used to analyze the Pearson correlation coefficient between the expression of the TGF-*β* signal regulator and other mRNAs. We used the Database for Annotation, Visualization and Integrated Discovery (DAVID) for the GO- and KEGG-enriched analysis and annotation database to comprehensively explore the potential biological significance of the list of genes of interest. The clusterProfiler software package of R software was used to visualize the enrichment results according to the *P* value (*P* < 0.05). In order to reveal the relationship between TGF-*β* signal regulators, we use the STRING database (https://string-db.org/) to build a PPI network [17].

The article "Comprehensive Analysis of the Expression of TGF-β Signaling Regulators and Prognosis in Human Esophageal Cancer" was published in 2021. Journal: Comput Math Methods Med.

### 2.4. Kaplan-Meier Plotter Database

The Proc software package [18] in the R software was used to analyze the ROC curve to explore the sensitivity and specificity of TGF-*β* signal regulators in EC. The Kaplan-Meier plotter (https://kmplot.com/) [19] is a database including microarray and TCGA gene expression data, which was used to analyze the correlation between TGF-*β* signal regulator expression and survival status in EC [20].

## 3. Results

### 3.1. Prognostic Relevance of Genomic Alterations in Patients with EC

In order to identify key pathways involved in regulating the progression of ESCC, we determined the prognosis of genomic alterations in multiple pathways using TCGA esophageal adenocarcinoma datasets, including TGF-beta, survival and cell death, cell cycle, migration and invasion, DNA damage, NOTCH, KRAS, RTK, PI3K-AKT, ribosome, and angiogenesis. We found that patients with mutations in TGF-beta, survival and cell death, cell cycle, migration and invasion, DNA damage, and NOTCH demonstrated worse prognosis compared with patients without mutated signaling (Figure 1).

Of note, we observed that TGF-beta was most significantly associated with the overall survival time in EC. To further confirm the prognostic value of TGF-beta signaling, we analyzed the correlation between mutations in this signaling and disease-free survival time (Figure 2(a)), disease-specific survival time (Figure 2(b)), platinum overall survival time (Figure 2(c)), and platinum progression free survival time (Figure 2(d)). As expected, we found that patients with mutations in TGF-beta signaling were significantly associated with shorter survival time compared to that without these mutations.

### 3.2. Genetic Alteration Differences of TGF-*β* Signaling Regulators in EC Patients

Furthermore, genetic alteration of TGF-*β* signaling regulators in EC was analyzed using the cBioPortal database, which included 1443 patients from seven related studies. The mutation, amplification, and deep deletion were the most common types of alteration in different EC subtypes (Figure 3(a)). We also observed that TGF-*β* signaling regulators were altered in 19% of EC patients (254/1354) (Figure 3(b)). The mutation rates of TGF-*β* signaling regulators for EC ranged from 0.8% to 12% for individual genes (SMAD4, 12%; SMAD7, 5%; ACVR2A, 6%; TGFBR2, 5%; BMP7, 5%; BMP5, 4%; BMP15, 4%; and BMPR2, 4%) (Figure 3(c)).

The article "Comprehensive Analysis of the Expression of TGF-β Signaling Regulators and Prognosis in Human Esophageal Cancer" was published in 2021. Journal: Comput Math Methods Med.

### 3.3. Relative Transcriptional Expression of TGF-*β* Signaling Regulators in EC Patients

Comparison of the RNA levels of TGF-*β* signaling regulators in EC and noncancer samples showed that RNA levels of ZFYVE9, BMPR1B, TGFB3, TGFBRAP1, ACVRL1, TGFBR2, SMAD4, SMAD7, ACVR2A, BMPR1A, SMAD9, and TGFBR3 were significantly downregulated in EC tumor samples compared to normal samples; however, ACVR1 and SMAD1 were upregulated in EC samples (Figure 4).

### 3.4. Diagnostic Value of TGF-*β* Signaling Regulators for Distinguishing EC Patients

To investigate the prognostic value of TGF-*β* signaling regulators in EC, we applied a ROC curve analysis using TCGA database (Figure 5). ROC analysis of TGF-*β* signaling regulators revealed that these regulators had high diagnostic value for distinguishing EC from normal individuals, including ACVR1 (0.7720), ACVRL1 (0.6865), ACVR2A (0.7789), SMAD1 (0.7219), SMAD7 (0.7356), SMAD4 (0.8550), SMAD9 (0.8349), BMPR1A (0.6791), BMPR1B (0.7681), TGFBRAP1 (0.8123), TGFBR2 (0.8354), TGFBR3 (0.8914), TGFB3 (0.7381), and ZFYVE9 (0.7553),

### 3.5. The Dysregulation of TGF-*β* Signaling Regulators Correlated with Longer Survival Time in EC

Our results showed upregulation of ACVR1, TGFBR3, TGFBRAP1, BMPR1A, SMAD4, and TGFBR2 associated with a short overall survival time in patients with EC (Figure 6).

### 3.6. Construction of the Protein-Protein Interaction Network Regulated by Hub TGF-*β* Signaling Regulators in EC

In order to investigate the potential mechanism of TGF-*β* signaling regulators in EC, we applied coexpression network analysis using the cBioPortal database and PPI network using the STRING database in ESCC. The correlation among ACVR1, ACVRL1, ACVR2A, SMAD1, SMAD7, SMAD4, SMAD9, BMPR1A, BMPR1B, TGFBRAP1, TGFBR2, TGFBR3, TGFB3, and ZFYVE9 is shown in Figure 7. The results showed that these hub genes could be divided into two subclasses, including subclass 1 (ACVR1, SMAD1, ZFYVE9, BMPR1B, and TGFB3) and subclass 2 (TGFBRAP1, ACVRL1, TGFBR2, SMAD4, SMAD7, ACVR2A, BMPR1A, SMAD9, and TGFBR3). The coexpressed genes with Spearman′s correlation > 0.8 were selected as the potential targets of hub genes in ESCC. The PPI network is shown in Figure 6. Based on PPI network analysis, we revealed several key targets of TGF-*β* signaling regulators in EC, including KDR, ACVR2A, PRRX1, ACVRL1, TGFBRAP1, GDF6, BMPR1B, ENG, CD, TGFBR2, SMAD4, SMAD7, FN1, SMAD1, ZFYVE9, ACVR1, TGFB3, VWF, SMAD9, BMPR1A, and TGFBR3.

The article "Comprehensive Analysis of the Expression of TGF-β Signaling Regulators and Prognosis in Human Esophageal Cancer" was published in 2021. Journal: Comput Math Methods Med.

### 3.7. Functional Enrichment Analysis of TGF-*β* Signaling Regulators

To investigate the functional roles in EC, we constructed the correlation between the expression of TGF-*β* signaling regulators, PPI network, GO analysis, and KEGG enrichment analysis (Figure 8). GO analysis showed that ACVR1, SMAD1, ZFYVE9, BMPR1B, and TGFB3 were related to regulating cell adhesion, extracellular matrix organization, collagen fibril organization, endodermal cell differentiation, angiogenesis, negative regulation of chondrocyte differentiation, extracellular matrix disassembly, integrin-mediated signaling pathway, and wound healing. And subclass 2 was related to regulating angiogenesis, cell adhesion, extracellular matrix organization, positive regulation of GTPase activity, signal transduction, PI3K signaling, Rho signal transduction, calcium ion transport, leukocyte migration, vasculogenesis, and peptidyl-tyrosine phosphorylation.

KEGG analysis showed that ACVR1, SMAD1, ZFYVE9, BMPR1B, and TGFB3 were related to regulating proteoglycan in cancer, focal adhesion, tight junction, PI3K-Akt signaling pathway, cell adhesion molecules (CAMs), Rap1 signaling pathway, osteoclast differentiation, and Hippo signaling pathway. And subclass 2 was related to regulating cell adhesion molecules (CAMs), Rap1 signaling, cGMP-PKG signaling, PI3K-Akt signaling pathway, calcium signaling, focal adhesion, Ras signaling, platelet activation, and *Staphylococcus aureus* infection.

## 4. Discussion

Previous studies had revealed that multiple oncogenetic pathways were related to the tumorigenesis and development of EC, such as TGF-beta, survival and cell death, cell cycle, migration and invasion, DNA damage, NOTCH, KRAS, RTK, PI3K-AKT, ribosome, and angiogenesis signaling. For example, in a normal esophagus, NOTCH regulates the development of the esophageal squamous epithelium [21]. In ESCC, NOTCH plays either a tumor suppressive or an oncogenetic role [21]. Activation of KRAS induces the AKT-mTOR or RAF-ERK-pathways, which have an important role in modulating tumor microenvironment in EC [22]. Angiogenesis has a fundamental role in cancer growth and metastasis [23]. In EC, increased angiogenesis regulator expression was reported to be related to worse response and prognosis of EC. In this study, as far as we know, we used various large databases including TCGA, GEO, STRING, and Kaplan-Meier plotter, for the first time to analyze the level, gene changes, and functions of TGF-*β* signal regulators in patients with esophageal cancer. Our results showed that the TGF-*β* signal plays an important role in the diagnosis of EC. ROC analysis showed that most TGF-*β* signal regulators have high diagnostic value in distinguishing EC from normal patients. KM analysis showed that ACVR1, TGFBR3, TGFBRAP1, BMPR1A, SMAD4, and TGFBR2 were positively correlated with OS prolongation. In addition, all TGF-*β* signal transduction regulators are closely related to multiple biological processes, including cell adhesion, extracellular matrix tissue, collagen catabolism, and PI3K signaling. In short, the members of TGF-*β* signal regulators can be potential biomarkers for the prediction of treatment and prognosis of EC.

The article "Comprehensive Analysis of the Expression of TGF-β Signaling Regulators and Prognosis in Human Esophageal Cancer" was published in 2021. Journal: Comput Math Methods Med.

More and more evidences indicate that TGF-*β* plays a key role in tumor cells and switches its function between tumor suppression and tumor promotion phenotypes [24]. For instance, TGF-*β* could arrest the cell cycle via CREB to mediate the histone acetylation of PAI-1 in a p53/Smad-dependent manner [25]. In addition, TGF-*β* can activate FoxO1 to induce the expression of p21cip1 to induce the G0/G1 arrest [11]. However, the role of the TGF-*β* factor in esophageal squamous cell carcinoma needs further study. Compared with TGF-*β*-mutant patients, we did find a worse prognosis in TGF-*β*-wild-type patients. In addition, we found that patients with TGF-*β* signaling mutations were significantly associated with shorter disease-free survival, disease-specific survival time, platinum overall survival time, and platinum progression-free survival time. Further analysis showed that ZFYVE9, BMPR1B, TGFB3, TGFBRAP1, ACVRL1, TGFBR2, SMAD4, SMAD7, ACVR2A, and BMPR1AEC patients had significantly lower expression, while ACVR1 and SMAD1 were expressed higher in EC than in normal samples. Thus, we showed that TGF-*β* regulators have high diagnostic capacity in distinguishing EC patients from healthy donors. To further clarify the genetic alteration of TGF-*β* signaling regulators, we analyzed the cBioPortal database and found that the percentages of genetic alterations in TGF-*β* signaling regulators for EC varied from 0.8 to 14% for individual genes.

Of note, our results showed upregulation of ACVR1, TGFBR3, TGFBRAP1, BMPR1A, SMAD4, and TGFBR2 associated with a short overall survival time in patients with EC. ACVR1 is an activin type I receptor including 509 amino acids [26]. The ACVR1 was found to be expressed in multiple human tissues and cell lines using RNA sequencing data. ACVR1 is a member of the BMP/TGF*β* receptor family [26]. ACVR1 forms a heterotetrameric receptor complex with BMPR2, ACVR2A, and ACVR2B [27]. When the signaling was activated, the type I receptor is trans-phosphorylated by the type II receptor. As a result, the kinase domain of the ACVR1 is activated and then phosphorylated the Smad1/5/8 protein [28]. In addition to the typical Smad signaling pathway, ACVR1 can also activate noncanonical signaling. New research shows that ACVR1 plays an important role in human cancer. For example, constitutively active mutants of ALK2 have been identified as the cause of FOP and were related to DIPG progression via modulating BMP signaling [29]. In pancreatic cancer, ACVR1 was found to regulate the stem cells and tumorigenicity of pancreatic cancer cells [30]. Deregulated ACVR1 was reported to be related to gastric cancer progression [31]. ACVR1 is significantly increased in esophageal tumors. In ESCC, the increase in the number of repeated copies of ACVR1 and the corresponding transcriptional overexpression are associated with the survival rate of patients with ESCC. In ESCC, TGFBR3 is an independent unfavourable prognostic marker and positively correlated with Ki-67 [32]. The key roles of SMAD4 in ESCC had been demonstrated in several previous reports. For example, Smad4 loss is associated with an increased propensity for disease recurrence and poor survival in EC, and Smad4 protein level was correlated with the depth of invasion of ESCC [33]. Smad7 is an inhibitory factor of the TGF-beta superfamily which was reported to be inversely correlated with depth of invasion of EC [34]. Our study for the first time comprehensively analyzed the prognostic value of these genes in EC.

The article "Comprehensive Analysis of the Expression of TGF-β Signaling Regulators and Prognosis in Human Esophageal Cancer" was published in 2021. Journal: Comput Math Methods Med.

To investigate the potential mechanism of TGF-*β* signaling regulators in EC, we applied coexpression network analysis using the cBioPortal database and PPI network using the STRING database in ESCC. The results showed that these hub genes could be divided into two subclasses, including subclass 1 (ACVR1, SMAD1, ZFYVE9, BMPR1B, and TGFB3) and subclass 2 (TGFBRAP1, ACVRL1, TGFBR2, SMAD4, SMAD7, ACVR2A, BMPR1A, SMAD9, and TGFBR3). Subclass 1 was involved in regulating cell adhesion, wound healing, PI3K-Akt signaling pathway, and Hippo signaling pathway. Of note, several previous studies had indicated that the hub genes in subclass 1 were related to the regulation of these signalings. For example, the activation of the intracellular BMP-Smad1/5 pathway regulated the expression of matrix macromolecules aggrecan and collagen II [35]. Subclass 2 was involved in regulating angiogenesis, cell adhesion, cGMP-PKG signaling, and PI3K-Akt signaling. Emerging studies demonstrated that the abnormal regulation of these signalings was observed in multiple tumors and related to tumor initiation and metastasis [36]. For example, the Hippo coactivator YAP1 mediates EGFR overexpression and confers chemoresistance in EC [37]. Targeting the Hippo coactivator YAP1 through BET bromodomain inhibition could suppress EC growth [38]. Of note, various studies had indicated that TGF-*β* signaling was cross talked with these signalings in human cancers. For example, TGF-*β* upregulates the translation of USP15 via the PI3K/AKT pathway to promote p53 stability [39]. PI3K/mTORC2 could regulate TGF-*β*/activin signalings by modulating Smad2/3 activity [40]. In triple negative breast cancer, TGF-*β* promotes noncanonical PI3K/Akt signaling by reducing PTEN [41]. In addition, TGF-*β* targets the Hippo pathway scaffold RASSF1A to facilitate YAP/SMAD2 nuclear translocation [42]. TGF-beta synergizes with defects in the Hippo pathway to stimulate human malignant mesothelioma growth [43]. Therefore, we hypothesized that the mechanism of the TGF-*β* signal regulator is to induce tumorigenesis and development by regulating these pathways. This provides new ideas for the diagnosis and treatment of EC.

The article "Comprehensive Analysis of the Expression of TGF-β Signaling Regulators and Prognosis in Human Esophageal Cancer" was published in 2021. Journal: Comput Math Methods Med.

Inevitably, this study had several limitations. First, most of the findings in this study were obtained using public databases. The biological functions of TGF-*β* regulators were unclear, and more experimental validation is needed to further confirm their functional importance in the EC. Second, TCGA database was used in this study. Further studies integrating multiomics datasets might strengthen the findings of this study. Third, the clinical information of the patients was limited. Thus, collecting more clinical samples to confirm the expression and mutation profile of TGF-*β* regulators is still needed.

## 5. Conclusions

In conclusion, TGF-*β* signal regulators are abnormally expressed in EC. The high expression of ACVR1, TGFBR3, TGFBRAP1, BMPR1A, Smad4, and TGFBR2 is positively correlated with prolongation of OS. These genes play a key role in EC and improve the survival rate and prognosis of the EC marker of accuracy.

## Figures and Tables

**Figure 1:** Prognostic relevance of genomic alterations of TGF-*β* signal regulators in human cancers. (a–k) The prognosis of genomic alterations in multiple pathways was determined using TCGA esophageal adenocarcinoma datasets, including TGF-beta (a), survival and cell death (b), cell cycle (c), migration and invasion (d), DNA damage (e), NOTCH (f), KRAS (g), RTK (h), PI3K-AKT (i), ribosome (j), and angiogenesis (k).

**Figure 2:** The correlation between mutation in TGF-*β* signal regulators and survival time in EC. (a–d) We analyzed the correlation between mutations in the TGF-*β* signal and disease-free survival time (a), disease-specific survival time (b), platinum overall survival time (c), and platinum progression-free survival time (d).

**Figure 3:** Genetic alteration differences of TGF-*β* signaling regulators in EC patients. (a) The genetic alteration of TGF-*β* signaling regulators in EC patients. (b) The mutation, amplification, and deep deletion were the most common types of alteration in different EC subtypes. (c) The hotspot mutations of SMAD2, SMAD7, ACVR2A, TGFBR2, and SMAD4.

The article "Comprehensive Analysis of the Expression of TGF-β Signaling Regulators and Prognosis in Human Esophageal Cancer" was published in 2021. Journal: Comput Math Methods Med.

**Figure 4:** Relative transcriptional expression of TGF-*β* signaling regulators in EC patients. (a) Heatmap showed the comparison of the RNA levels of TGF-*β* signaling regulators in EC and noncancer samples. (b) ZFYVE9, BMPR1B, TGFB3, TGFBRAP1, ACVRL1, TGFBR2, SMAD4, SMAD7, ACVR2A, BMPR1A, SMAD9, and TGFBR3 were significantly downregulated in EC tumor samples compared to normal samples; however, ACVR1 and SMAD1 were upregulated in EC samples.

**Figure 5:** Diagnostic value of TGF-*β* signaling regulators for distinguishing EC patients. (a–n) ROC analysis of TGF-*β* signaling regulators revealed that these regulators had high diagnostic value for distinguishing EC from normal individuals, including ACVR1 (a), ACVRL1 (b), ACVR2A (c), SMAD1 (d), SMAD7 (e), SMAD4 (f), SMAD9 (g), BMPR1A (h), BMPR1B (i), TGFBRAP1 (j), TGFBR2 (k), TGFBR3 (l), TGFB3 (m), and ZFYVE9 (n).

**Figure 6:** The dysregulation of TGF-*β* signaling regulators correlated with longer survival time in EC. (a–f) Our results showed upregulation of ACVR1 (a), TGFBR3 (b), TGFBRAP1 (c), BMPR1A (d), SMAD4 (e), and TGFBR2 (f) associated with a short overall survival time in patients with EC.

**Figure 7:** Construction of the protein-protein interaction network regulated by hub TGF-*β* signaling regulators in EC. (a) The correlation among ACVR1, ACVRL1, ACVR2A, SMAD1, SMAD7, SMAD4, SMAD9, BMPR1A, BMPR1B, TGFBRAP1, TGFBR2, TGFBR3, TGFB3, and ZFYVE9 was shown. (b) The PPI network was constructed to show the interaction among KDR, ACVR2A, PRRX1, ACVRL1, TGFBRAP1, GDF6, BMPR1B, ENG, CD, TGFBR2, SMAD4, SMAD7, FN1, SMAD1, ZFYVE9, ACVR1, TGFB3, VWF, SMAD9, BMPR1A, and TGFBR3.

**Figure 8:** Functional enrichment analysis of TGF-*β* signaling regulators: (a, b) the GO and KEGG analysis of subclass 1 genes; (c, d) the GO and KEGG analysis of subclass 2 genes.

## Data Availability

The expression profile of the TGF-*β* signal regulator is retrieved from TCGA-ESCA database, and the clinicopathological information of EC patients is also downloaded from this database.
